The article "Causes of Emergency Bleeding after Nonsurgical Periodontal Therapy in Adult Periodontitis Patients: A Retrospective Analysis" was retracted in 2023. Reasons: signs of a paper mill; suspected computer-generated content; unreliable results or conclusions; concerns about the data.

# Causes of Emergency Bleeding after Nonsurgical Periodontal Therapy in Adult Periodontitis Patients: A Retrospective Analysis

**DOI:** 10.1155/2022/1579574

**Published:** 2022-03-29

**Authors:** Fei Lu, Gang-Gang Qi, Wen Fang, Xin Zhang, Jing Zhou, Xue-Fen Yu, Xiao-Jun Li

**Affiliations:** Stomatology Hospital, School of Stomatology, Zhejiang University School of Medicine, Zhejiang Provincial Clinical Research Center for Oral Diseases, Key Laboratory of Oral Biomedical Research of Zhejiang Province, Cancer Center of Zhejiang University, Hangzhou 310006, China

## Abstract

**Background:**

Emergency gingival uncontrollable bleeding after nonsurgical periodontal therapy (NSPT) could be caused by a variety of factors; local oral factors are the main cause of gingival bleeding in most patients. Because the doctor will do a good job of evaluating the patient's physical condition before nonsurgical periodontal therapy. This study is subjected to evaluate the possible factors associated with emergency uncontrollable bleeding within 24-48 hours after NSPT. *Material and Methods*. A total of fifty-eight patients with emergency bleeding after NSPT in the past four years were enrolled. The related factors in patients, such as age, gender, clotting function, systemic diseases, and baseline periodontitis severity, were analyzed. The site-related factors, such as tooth type, tooth distribution, and alveolar bone resorption at the bleeding site, were compared. The possible relationship of the parameters to the causes of emergency bleeding with NSPT was also evaluated.

**Results:**

Gingival bleeding after NSPT was registered. In this retrospective study, a total of 58 patients were selected. There were 29 males and 29 females, aged from 20 to 67 years old, with an average age of 35.21 ± 10.09 years. Among them, 8.6% were over 50 years old, and 91.4% were under 50 years old. Completed evaluations were performed in 15.5% gingivitis and 84.5% periodontitis. The causes of emergency bleeding after nonsurgical periodontal therapy in this study were residual subgingival calculus or granulation tissue in 63.79% of cases: severe gingival inflammation, 29.32%; gum trauma, 3.45%; and poor compliance, 3.45%. The therapy method before bleeding includes supragingival scaling accounted for 72.4% and subgingival scaling accounted for 27.6%. 23 cases of horizontal absorption at the bleeding site accounted for 39.66%, and 35 cases of angular absorption accounted for 60.34%. Bleeding of maxillary posterior teeth accounted for 34.48%; mandibular anterior teeth accounted for 15.52%; mandibular anterior teeth accounted for 8.62%; and mandibular posterior teeth accounted for 18.97%; multiple sites accounted for 22.41%; eliminating residual subgingival calculus and granulation tissue were the main and most effective hemostatic methods, 86.21%.

**Conclusion:**

Residual subgingival calculus or granulation tissue and severe gingival inflammation were the main causes of emergency gingival bleeding after nonsurgical periodontal therapy. Severe gingival inflammation causing emergency bleeding was more common in maxillary posterior teeth areas. Angular alveolar bone resorption was more likely to cause bleeding than horizontal resorption. Careful debridement of residual subgingival calculus and granulation tissue was the main hemostatic method.

## 1. Introduction

Periodontal disease is a major inflammatory disease of the gums and bone that surround and support the teeth. It is the leading cause of tooth in adults. It is the main cause of tooth loss in adults. Advanced periodontitis can adversely impact the quality of life and the physical and mental health of patients. Periodontal disease has been causally linked to systemic diseases, such as cardiovascular disease and Alzheimer's disease [1–3]. In China, the prevalence of periodontal disease has shown an obvious increasing trend. The fourth national oral epidemiological survey showed that the rate of dental calculus detection in adults was as high as 96.7% [4].

Periodontitis is a bacterial inflammatory disease caused by dental plaque. The goal of the periodontitis therapy is to address gingival inflammation and restore periodontal health. Periodontal therapy always begins with nonsurgical periodontal therapy (NSPT) [5]. NSPT is engaged to preserve, improve, and maintain natural dentition [6], including by controlling (reducing/eliminating) the subgingival biofilm and calculus through manual subgingival instrumentation and follow-up in all periodontitis patients, irrespective of the disease stage, for all teeth with loss of periodontal support and/or periodontal pocket formation [7].

There are almost rarely studies on emergency bleeding after nonsurgical periodontal therapy. The study of Sumra et al. [8] mentioned that laser can promote wound healing in the early acute phase after mechanical debridement of periodontal nonsurgical treatment. Dilsiz and Sevinc [9] showed that the Nd : YAG laser appeared to significantly reduce instrument trauma while having a hemostatic effect, and a photoablation using a *λ* 810 nm diode laser was reported in Giannelli et al. [10] to specifically induce gingival microvascular constriction, preventing bleeding and producing a clean surgical area; Shiloah et al. [11] study show that daily intake of 325 mg ASA after scaling and root planing improves outcomes in smokers without increasing gingival bleeding tendency. The study of Ding et al. [12] selected 69 patients with chronic periodontitis complicated with coronary heart disease as the experimental group (drug group, group A) and the control group (discontinuation group, group B), including 20 patients with chronic periodontitis complicated with coronary heart disease who discontinued the drug for one week. A control group of 50 patients with chronic periodontitis (group C) was set up for 1 week. Three groups underwent pocket exploration and underwent supragingival scaling, subgingival scaling, and root planing. For postoperative observation of local bleeding, after 30 minutes of periodontal mechanical treatment, 5 cases in group A, 1 case in group B, and 1 case in group C had active bleeding, and some hemostatic measures were taken (containing oxidized cellulose into the periodontal pocket, compressed with gauze, and sutured). Bleeding was successfully stopped by Nd : YAG laser 60 minutes after operation.

With increasing public oral health awareness, an increasing number of patients are receiving periodontal therapy. The most common symptom of periodontal disease is gingival bleeding, and gingival bleeding is often observed in the therapy process. In a few cases, gingival bleeding and other complications will occur after therapy, which has an important impact on the daily life and mental health of patients [13]. Therefore, it is of vital importance to determine the cause of gingival bleeding after periodontal therapy and to address it accurately and promptly [14, 15]. Patient-related factors of such bleeding include severe gingival inflammation, coagulation disorder, and residual subgingival calculus. The aim of this retrospective study was to determine the causes and associated factors of bleeding in 58 patients after NSPT. A better understanding of these epidemiological factors will advance the management of periodontal disease from therapy to prevention.

## 2. Materials and Methods

### 2.1. Materials

This study was approved by Stomatology Research Ethics Committee of the Affiliated Stomatology Hospital (No. 2021-32) of Zhejiang University School of Medicine. All data were obtained retrospectively from therapy records. The patients involved had provided permission in advance for the analysis and publication of their treatment data. This retrospective study is based on patient data extracted from a computerized database from March 2017 to January 2021. All the records were analyzed thoroughly, and data concerning the patient's age, gender, diagnosis, coagulation function, history of systemic disease, and panoramic X-ray images were collected.

### 2.2. Methods

A total of 58 patients with emergency bleeding after NSPT were selected for this retrospective analysis in adult periodontitis patients. Among them, 50% males and 50% females, ranging in age from 20 to 67 years, with an average age of 35.21 ± 10.09 years. After clinical examination, all patients were diagnosed with active gingival bleeding requiring clinical hemostasis.

Senior attending stomatologists clinically examined the patients; then, the possible causes of gingival bleeding were analyzed, and treatment for hemostasis was performed. Hemostatic methods included local compression, debridement, periodontal subgingival curettage, suturing, and medication.

### 2.3. Statistical Analysis

The data of this study were extracted from the patients' files and entered into a computerized database anonymously.

## 3. Results

A total of 58 patients with emergency bleeding after NSPT were treated between March 2017 and January 2021. The proportion of men was 50% and that of women was 50%. The mean age at the time of treatment during the study period ranged from 20 to 67 years. 8.6% were over 50 years old, and 91.4% were under 50 years old. Gingival bleeding after NSPT was registered. The treatment method before bleeding includes supragingival scaling accounted for 72.4% and subgingival scaling accounted for 27.6%. Gingival bleeding after NSPT was registered. Completed evaluations were performed in 15.5% gingivitis and 84.5% periodontitis of cases. Extract data summary is in Table 1.

### 3.1. Causes of Uncontrollable Bleeding

During the reviewed period between March 2017 and January 2021, there were 58 patients with emergency periodontal bleeding after NSPT. Among the causes of bleeding, residual subgingival calculus or granulation tissue accounted for 63.79% of cases. Deep periodontal pockets, crowded dentition or difficulty scaling posterior teeth area, and severe periodontitis all contributed to residual subgingival calculus or granulation tissue. Additionally, severe gingival inflammation was observed in 29.31% of patients and poor compliance in 3.45% of patients, Treatment-associated trauma accounted for 3.45% of cases. In gingivitis and periodontitis patients, subgingival calculus or granulation residue was the most common causes of emergency bleeding after NSPT (Table 2).

### 3.2. Distribution of Bleeding Sites

Bleeding occurred more often in the mandibular anterior teeth than in the maxillary anterior teeth, and the bleeding was more serious in maxillary posterior teeth than in mandibular posterior teeth. Severe gingival inflammation causing emergency bleeding was more common in maxillary posterior teeth areas (Table 3).

### 3.3. Type of Alveolar Bone Resorption at Bleeding Site

The results of the present study show that 23 cases of horizontal absorption at the bleeding site, accounting for 39.66%, and 35 cases of angular absorption, accounting for 60.34%.

Angular alveolar bone resorption was more likely to cause bleeding than horizontal resorption. (Table 4, Figures 1–3).

### 3.4. Haemostatic Methods

According to this retrospective analysis, eliminating residual subgingival calculus and granulation tissue were the main and most effective hemostatic methods (Table 5).

## 4. Discussion

This retrospective analysis evaluated causes of emergency bleeding after NSPT in the past four years. This study was conducted to determine the association of the severity of gingival bleeding with age and sex and whether it tends to be site-specific. Meanwhile, we investigated whether the type of alveolar bone resorption was associated with gingival bleeding.

Routine blood and coagulation function examinations before NSPT can be used to screen for patients with systemic disease affecting the blood and abnormalities in coagulation function. If such patients are treated directly, they will often exhibit severe bleeding symptoms, and due to the combination of systemic factors, the effect of hemostatic treatment is poor. Therefore, preoperative evaluations of the blood test results and medical history are also very important. With the improvement of Chinese people's living standards and changes in dietary habits, the elderly population is increasing annually, and the incidence and number of cardiovascular diseases and the number of patients receiving anticoagulation therapy are also increasing year by year. Due to the risk of bleeding, it was previously suggested that the use of anticoagulant drugs should be stopped for a few days before surgery to restore coagulation function. However, this approach resulted in an increased risk of thrombosis. In view of the risk of thrombosis after the discontinuation of anticoagulant drugs in patients with invasive oral diagnostic and treatment procedures, Wahl conducted a retrospective study on the risk of thrombosis after the discontinuation of antiplatelet drugs in 324 such patients; among them, 17 patients (5%) developed thrombosis complications [16]. In the case of antiplatelet therapy, some results suggest that continued aspirin treatment does not increase the risk of bleeding after tooth extraction [17, 18]. The discontinuation of antiplatelet drug use was associated with a 3.4-fold increased risk of ischemic shock [19]. Studies have shown that systemic aspirin administration can cause bleeding of the gums [20]. However, some patients who used anticoagulant drugs for a long time such as activated partial thromboplastin time (APTT) and prothrombin time (PT) were not significantly changed in indexes of coagulation function, which is also consistent with other studies. Therefore, as long as these patients have no obvious abnormalities in coagulation function indexes, they can also undergo routine periodontal treatment without suspending drug use to avoid the increased risk of thrombosis. However, treating such patients requires procedures to be performed gently and carefully in subzones, followed by observation for more than 30 minutes after treatment to identify bleeding symptoms. If the patient has any bleeding symptoms, the patient should see a doctor immediately for timely medical treatment. In this study, a total of 4 patients were receiving anticoagulant medication. However, the coagulation indexes of these 4 patients were all within the normal ranges. Anticoagulant drug use did not increase the difficulty of hemostasis in these patients compared with that in other patients.

In this study, it was found that poor patient compliance and improper management were also important causes of postoperative gingival bleeding. It is generally believed that oral hygiene instruction (OHI) in periodontal treatment mainly includes the following: (1) informing the patient of the importance of oral hygiene in the process of periodontal treatment, (2) developing appropriate measures for the patient to maintain oral health, (3) assessing the patient's ability to perform these measures as planned, and (4) ensuring that the patient can carry out the medical orders for OHI for a long time. Tonetti et al. [21] believe that OHI is an important intervention measure throughout the process of treating periodontitis. The awareness of medical orders after treatment should also be promoted and after treatment, including removing plaque around the teeth, noticing the original state of the teeth and gums; however, some patients do not adapt or do not stop using their tongue to lick the gums or make clicks. After the treatment of these patients, bleeding may occur, necessitating gargling or even wiping the gums with a paper towel. On the other hand, the mixture of blood from gingival bleeding with saliva in the mouth often gives patients the impression of a very large amount of bleeding, resulting in psychological distress. These behaviours could lead to more postoperative gingival bleeding. Therefore, patients should be provided with specific and detailed postoperative medical advice to avoid these situations.

NSPT has been proved to improve the level of clinical attachment and effectively reduce the probing pocket depth [22, 23]. Therapy includes oral hygiene instruction, subgingival scaling, and root planing [5]. Gingival bleeding is the most common complication after supra- and subgingival curettage and the most common symptom in periodontal emergency departments [24]. This study found that the site of gingival bleeding was specific to the site of NSPT. In most cases, the cause of emergency bleeding was residual subgingival dental calculus or severe gingival inflammation. This may be related to deep periodontal pockets and molar furcation involvement. Some studies [25, 26] have shown that the treatment success rate of single root is higher than that of molar. In these studies, the results depend on the type of tooth, root bifurcation disease, and the severity of periodontitis. Other authors [27, 28] have considered this may be related to the anatomy of teeth. Multiroot teeth have difficulties in periodontal treatment.

There were 50 patients with periodontitis and 8 patients with gingivitis in this study. The findings and results of this study show that the most common treatment before gingival bleeding was ultrasonic scaling. Ultrasonic scaling was performed in 34 patients with periodontitis, and gingival inflammation and residual subgingival calculus and granulation tissue were identified as causes of bleeding. In patients with severe periodontitis, the area of ulceration in the periodontal pocket can reach 72 cm^2^, and there is much inflammatory granulation tissue in the inner wall of the periodontal pocket. The traumatic effect of the residual calculus in the inner wall of the periodontal pocket after curettage can lead to spontaneous bleeding of the gums. In this case, the sharp residual subgingival calculus and granulation tissue can cause bleeding symptoms.^20^ Residual calculus in the subgingiva can irritate periodontal tissue or puncture small blood vessels, causing bleeding. Therefore, in the course of treatment, careful exploration should be performed to avoid leaving residual subgingival calculus. In addition, a treatment plan should be made according to the degree of periodontal inflammation and the general condition of the patient [29]. If the periodontal inflammation is serious, subgingival treatment should be performed step by step after the gingival inflammation is partly relieved. During treatment, application of the ultrasonic device at an excessive power or to an excessive degree should be avoided, as this will contribute to the gingival trauma and thereby increase the risk of postoperative bleeding.

The results of the present study also show that angular alveolar bone resorption was more likely to cause bleeding after NSPT. This may be related to the characteristics of angular absorption. In angular reportion, calculus in the periodontal pocket calculus is more difficult to remove completely, and it is easy to leave residual dental calculus and granulation tissue. No similar reports have been found. Further large-sample studies are needed to confirm these conclusions.

There are some limitations in our study. The data collected did not include the patient's smoking history and baseline of periodontal pocket. In this retrospective analysis, digital electronic medical is in its infancy, and there are many patients and doctors have great pressure to receive them. Digital electronic medical records are not perfect, so it can not provide more population information for this study. The findings of this retrospective analysis need to be further investigated in a larger sample for verification. In the present analysis, many factors have been considered by the authors before the outcome of treatment. Therefore, the originality of this study can be considered to be limited.

## 5. Conclusion

Within the limitations of this retrospective analysis, the authors conclude that residual subgingival calculus or granulation tissue and severe gingival inflammation were the main causes of emergency gingival bleeding after NSPT. In addition, a significant difference in emergency bleeding was observed according to the method of treatment before gingival bleeding and the type of alveolar bone resorption.

## Figures and Tables

**Figure 1:** 47 mesoangular absorption.

**Figure 2:** 26, 27 angular absorption.

**Figure 3:** 12 distal angular absorption.

**(a):** 

Age		Sex		Treatment method before bleeding	
≤50	>50	Male	Female	Supragingival	Ubgingival scaling

53(91.4%)	5(8.6%)	29(50%)	29(50%)	42(72.4%)	16(27.6%)

**Table:** (b) Following the table above

Periodontal condition		Hypertension		Clotting disorder	
Gingivitis	Periodontitis	Yes	No	Yes	No

9(15.5%)	49(84.5%)	4(6.9%)	54(93.1%)	17(29.3%)	41(70.7%)

**Table 2:** Causes of emergency bleeding after nonsurgical periodontal therapy.

Causes of emergency bleeding	*N* = 58 (%)	Gingivitis (%)	Periodontitis (%)
Subgingival calculus or granulation residue	37 (63.79)	7 (87.5)	30 (60)
Severe of gingivitis inflammation	17 (29.31)	1 (12.5)	16 (32)
Poor compliance	2 (3.45)	0	2 (4)
Gum trauma	2 (3.45)	0	2 (4)

**Table 3:** Distribution of bleeding teeth after nonsurgical periodontal therapy.

Bleeding site	*N* = 58	Percentage (%)
Maxillary anterior teeth	5	8.62
Mandibular anterior teeth	9	15.52
Maxillary posterior teeth	20	34.48
Mandibular posterior teeth	11	18.97
Multiple sites	13	22.41

**Table 4:** Type of alveolar bone resorption at bleeding sites.

Type of alveolar bone resorption	Bleeding	Percentage (%)
	58	100
Horizontal resorption	23	39.66
Angular resorption	35	60.34

**Table 5:** Hemostatic methods.

Hemostasis method	*N* = 58	%
Ultrasonic subgingival debridement	50	86.21
Debridement+hemostyptic	3	5.17
Debridement+periodontal dressing	2	3.45
Hemostasis by compression	3	5.17

## Data Availability

The data used to support the findings of this study are available from the corresponding author upon request.

## Abbreviations

NSPT: Nonsurgical periodontal therapy
APTT: Activated partial thromboplastin time
PT: Prothrombin time.
